# Research on Learning Evaluation of Online General Education Course Based on BP Neural Network

**DOI:** 10.1155/2021/3570273

**Published:** 2021-12-06

**Authors:** Zongbiao Zhang

**Affiliations:** Office of Academic Affairs, Zhejiang Shuren College, Hangzhou 310015, China

## Abstract

Network open curriculum provides a new solution for general education in local colleges and universities, which makes the network curriculum widely popularized and applied in colleges and universities. However, due to the lack of good curriculum learning evaluation, it is inconvenient for learners to choose. Therefore, this paper proposes to use the BP neural network model to evaluate the learning process of network general education course. Based on the course and user data provided by the existing platform, this paper constructs an online course learning evaluation model and studies the structure and effect relationship among learning experience, learning investment, and learning performance of ordinary online courses based on the preaging process product (3P) model and structural analysis method. Our research shows that curriculum quality is a key factor in analyzing and predicting learning results, which has a great impact on learning achievement. Learning experience is a direct factor affecting academic achievement. Learning experience, as an intermediary variable, indirectly affects e-learning performance. At the same time, it puts forward some suggestions to optimize the learning effect of ordinary online courses. On the one hand, the evaluation model provided in this paper can provide a reference for learners to select online courses; on the other hand, it can also be used as a supplement to the existing subjective evaluation model.

## 1. Introduction

General course aims in providing a broader and more comprehensive education for college students and enriches them with necessary knowledge and abilities for postgraduate practice. This concept originated from Europe, developed in the United States decades ago, especially after the Harvard committee established and published the “General Education in a Free Society” (the Harvard Redbook, 1945) [1, 2]. It caused an applauded response in the American higher education society and boomed around the world later. After the Chinese Economic Reform in 1978, the higher education in China started a progressive qualitative education reform and addressed the connection between vocational education and general education. Recently, colleges in China are exploring novelties and possibilities in general education theoretically and practically. Outstanding accomplishments were achieved, and some adapted general education models was established. These achievements have a significant impact in Chinese higher education [3].

Compared with first-class universities, regional colleges have some shared problems such as lacking faculty and staff, unbalanced course arrangement for different subjects, and setting up courses by number of students [4]. With the development of online open course, these problems are well relieved. Currently, there are more than 2000 universities, and more than 10 million students are using online learning platform in China. The online learning platform has become an important carrier for general education of regional college. However, challenges emerged with the succeeding of online teaching at the same time. For example, misunderstanding of course content during course selection, impure motivation in learning, imperfection of course assessment, assurance of course quality, marginalized course management, and plagiarisms. Based on a case study in our college, start from spring 2020, 400 modelized open general courses were offered for all students. Data for latest two years are given in Table 1. It is easy to find the “high selection rate-low complete rate-high excellent rate” pattern in Table 1. This led to questions on providing qualitative online general course. How was the students' learning experience in the online general course? How to accurately control learning performance and its key factors? How to optimize the learning performance? Many scholars considered learning experience, learning engagement as the major factors for online learning [5, 6]. As a result, this study was theoretically based on the Dr. Bigg's “presage-process-product” model. We applied the structural equation modeling analysis method and discussed the structure and effect between learning experience, learning engagement, and learning performance for online general course. We were also aiming at optimizing the online learning performance, improving the general education quality, and providing future considerations on online general course in China.

## 2. Method and Modeling

Biggs pointed out that the early variables include student's personality and learning experience, and process variables include learning engagement and feeling to the course content in the learning process [7]. Based on the 3P theory, we provide an online general course learning relationship model (Figure 1). Taking the online learning experience as the main factor in the presage stage, taking the online learning engagement and course content quality as main factors in the process stage, and taking the online learning performance as the key factor in the product stage, the interaction between different factors forms a dynamic model.

### 2.1. Variables in Presage

Presage variables determine the attitude and method of the learner which further determines the learning product. As the direct participant and experiencer, students who attend the online course are affected by various factors such as the perception and experience for learning process and product.

Online learning experience positivity influences the online learning performance. Study shows strong correlation for the online learning experience and individual specialties of the students [8]. The individual specialties usually include willingness and motivation of learning, self-regulation ability, and information attainments [9, 10].

In this case, we propose that H1-H2, online learning experience has positive effect on online learning engagement and online learning performance.

### 2.2. Variables in Process

Process variables in online learning are mainly discussing whether the learning method could satisfy the learner's experience and whether the online learning performance could reach the preset goals. Course content quality control is one of the key targets for the online learning management. Online learning engagement affects the learning quality greatly as well. Both of them affect the learning process significantly [11]. In this case, we investigated the online learning engagement and course quality as the major process variables.

Course content quality actively affects the online learning experience. Study shows the content and experience are in the relationship of demand and satisfaction [12]. Qualitative course content satisfies the learner with a higher learning experience, incites their mind and feeling, emotional, and positively gains them knowledge. Factors for online learning experience include online course anxiety, course content quality, perception of the usefulness of the course, flexibility of the course [13]. Course quality has positive impact on the online learning engagement. Study shows the interaction between learner and course content deeply reflects the degree of perception for learning engagement [14]. Modeling of online learning theory should focus on the positive learning experience and learning engagement concentration of the learner in an organic and unified information environment, paying attention to the thinking and interestingness of the content. Online course quality will have a positive impact on online learning performance. Research shows that appropriate course content is a key factor in the performance of teaching and online learning. Quality perception has a great impact on academic achievement. At the same time, the learning performance is directly affected by the perception of course value.

Online learning engagement has positive impact on online learning performance. Study shows increasing learner's learning engagement promote the learner's further in-depth processing, speculation, analysis reasoning, and argumentation of the learning content. It has significant impact on the learning performance as well [15–17]. Other classification research on the relationship between online learning engagement and performance in distance education shows positive relationship between online learning engagement and online learning performance in 60% of the learners [18].

Therefore, we assume (a) course content quality has positive effect on online learning experience, online learning engagement and online learning performance (H3-H5); (b) online learning engagement has positive effect on online learning performance (H6).

### 2.3. Variables in Product

Variables for learning product mainly include the performance and product of learner, they are directly affected by presage variables and process variables. Online learning performance, also called E-learning performance or digital learning performance, is both (a) learning grade and performance achieved by the learner, and (b) information literacy consciousness, knowledge and skill improvement, learning experience satisfaction [19], etc. Currently, comprehensive, systematic, and in-depth studies on online learning performance have been carried out internationally. Overall, low online learning performance, low online course quality has significant long-term impact on college education. It is theoretically and practically important to figure out the factors for online learning performance [20]. This study uses online learning performance as the course product variable. We have added requirements for student abilities and emotions considering the online general courses are basic, accommodating, and profound. For instance, through the online general courses, students have formed general sense abilities, positive emotion, and attitude. This outcome aligns with our goal and highlights characteristics of general education.

The variable relationship among learners, learning process variables, and learning performance is shown in Figure 2.

### 2.4. Implementation Process of the BP Neural Network

BP neural network, also known as back propagation neural network, its main working principle is to use machine learning to continuously iterate the training model, adjust the weight in the network structure, gradually optimize the model structure, make the error function decline along the negative gradient direction, and make the output value of the model constantly close to the expected value. The input layer described in this paper includes the following nodes: online learning experience, online learning engagement, course content quality, and online learning performance. The output layer has only label degree, that is, the output layer is one node. The number of nodes in the hidden layer is *l*, which is obtained through the analysis of training experiments.

In order to eliminate the influence of different dimensions among the four evaluation indicators: the number of course interaction, the number of course selection schools, the number of course selection and the number of viewers, the data are standardized. The index variables are mapped to [0,1] through normalization, and the formula is as follows:

(1) $$\begin{array}{c} p_{i}^{m}=\frac{P_{i}^{m}-P_{i\min}}{P_{i\max}-P_{i\min}}, \end{array}$$

where *i*=1,2,…, 4, *m*=1,2,…, 400, *P*_*i*max_ and *P*_*i*min_ are the maximum and minimum values in the *m*-th original data, and *p*_*i*_^*m*^ (*m*=400) is the normalized data. 80% of the data are randomly selected from the normalized data set as training data and the remaining 20% as test data.

Input the training data into the neural network, and the output value of the hidden layer can be obtained through equation (2), shown as follows:

(2) $$\begin{array}{c} l_{j}^{m}=\sum_{i=1}^{4}w_{ij}^{\left(z\right)}P_{i}^{m}+h_{j}^{\left(z\right)}, \end{array}$$

where *j*=1,2,…, *n*, *n* is the number of nodes in the hidden layer, *w*_*ij*_^(*z*)^ is the connection weight between the input layer and the hidden layer, and *h*_*j*_^(*z*)^ is the threshold of the hidden layer.

### 2.5. Construction of the BP Neural Network Model

In order to explore the internal relationship between different evaluation objects and indicators, the BP neural network model can be constructed based on the existing sample data. This paper will fully consider and reasonably determine the key factors such as the structure, algorithm, neuron number, and error accuracy of the network model and make the model have a certain generalization ability. The BP neural network model structure for analyzing the relationship among learners, learning process variables, and learning performance is shown in Figure 3.

Because the number of neurons in the input layer depends on the number of variables contained in the problem, this study involves learners, learning process variables, and learning performance. The output layer mainly depends on the research results. After comprehensive analysis and judgment, select the number of neurons in the output layer. The output of this study is the relationship among learning performance, learners and learning process variables. Therefore, this paper sets the number of neurons in the output layer to 1. From the above analysis, the BP neural network constructed in this paper contains only one hidden layer. Because the number of hidden layer neurons will directly affect the accuracy of network training, the number of neurons should be considered according to needs. If the number of hidden layer neurons is too small, it will greatly reduce the fault tolerance of the network model and the accuracy of sample recognition. If you set too many times, the network training time will be too long, and the fitting degree of the network model will be greatly improved, resulting in overfitting problems.

## 3. Research Design

### 3.1. Research Content

Based on previous research results and 3P model, this study empirically explored the structural and effect relationship among online general learning experience, engagement, and performance in regional undergraduate schools from the perspective of general education, to explore ways and methods of which promoting teaching quality of online general course. This study focuses on the following issues: (a) validation of the theoretical model of online learning experience, online learning engagement, course content quality, and online learning performance; (b) if validated, the effects among each factor in the model and the degree of effectiveness of the online general course.

### 3.2. Research Target

This study used convenience sampling on undergraduate students from five regional colleges in Zhejiang, China. We used the questionnaire survey method to collect relevant data and information. 685 questionnaires were successfully returned and analyzed. After screening by three standards: (1) no learning experience of online general course; (2) variable answers were all the same for variables; (3) answers for the variable items are missing, a total of 583 valid samples remained, with an effective rate of 85.11%.

Sample compositions are listed as follows:

  Male: 257 (44.1%), female: 326 (55.9%)
  Freshman: 162 (27.8%), Sophomore: 211 (36.2%)
  Junior: 139 (23.8%), senior: 71 (12.2%)
  Science and engineering: 189 (32.4%), literature/economics/financial/management: 154 (26.4%), agriculture and medicine: 78 (13.4%), art and edu: 92 (15.8%), law/history/philosophy: 70 (12%)
  Course attended: 1 course: 75 (12.9%); 2-3 courses: 125 (21.4%); 4-5 courses: 245 (42%); more than 5: 138 (23.7%).

### 3.3. Research Method

SPSS 25.0 was used for data descriptive statistics and correlation analysis. AMOS 24.0 was used to establish the structural equation model. Maximum likelihood estimation method was used to evaluate the fitness of the model. Relative path analysis was combined to define the model.

### 3.4. Research Tool

In this study, a scale was developed to measure students learning status by literature reviews and student interviews. The scale includes two parts: learner's basic information (4 items) and survey on online general course (35 items). Each item in the second part was designed from the Likert's five-point scale (1 = strongly disagree, 5 = strongly agree). As shown in Table 2, the survey items are mostly referred to domestic influencing factor scales for various studies on general education.

To guarantee reliability and validity of the model, we used T-test for project analysis; we adopted internal consistency method for reliability evaluation; we used factor analysis method for construct validity test; we deleted one item from the learning engagement subscale, kept 34 items; and we deleted latent variables with a loading less than 0.5. Finally, dimensionality reduction was performed by calculating variables to determine 4 latent variables and 28 observed variables.

## 4. Results and Discussion

### 4.1. Measurement Model Testing

SPSS25.0 was used to perform reliability and validity test on the measurement model. In the model's reliability test, as shown in Table 3, from the view of average value, each latent variable is higher than the theoretical median (3 point). This indicates that learner's evaluation tends to be positive. Further improvement in online learning engagement is expected. From the view of standard deviation, the fluctuation of online learning engagement is high. Cronbach's *α* value is greater than 0.7, which implies data are reliable with high confidence. All average variance extracted (AVE) values are greater than 0.5, and all combination reliability (CR) is greater than 0.8, which indicate that the inherent quality of latent variables is good, and convergent validity is ideal. As a conclusion, the reliability of this measurement model is good.

In the model's validity test, as shown in Table 4, this model passed Bartlett's test.KMO >0.8, *P* < 0.000, and passed the significance test. This indicates the latent variables are suitable for factor analysis. The factor loadings of the observed variables are all greater than 0.7, eigenvalues are greater than 3, and cumulative variance explained rates are greater than 70%. As a conclusion, the overall validity of the measurement model is good.

### 4.2. Structural Model Testing

AMOS24.0 was used for confirmatory test on the structural model. The result shows the fitting index of the model is good. *X*^2^/df = 2.859, RMSEA = 0.056, NFI = 0.868, RFI = 0.848, CFI = 0.903, IFI = 0.904, and TLI = 0.952. The discriminative validity test results for the structural model are shown in Table 5. The absolute values of the correlation coefficients of the observed variables are all less than 0.5 and are all less than the square root of the corresponding AVE. This indicates the model has an ideal discriminative validity.

### 4.3. Hypothesis Testing

This section uses hypothesis testing in the model to analyze the effect and relationship between course content quality, online learning experience, online learning engagement, and online learning performance. As shown in Table 6, course content quality has a significant positive impact on both online learning experience (*β* = 0.724, *P* < 0.001) and online learning performance (*β* = 0.507, *P* < 0.001), respectively, indicating that high-quality course content leads to high learning experience. This will not only help to improve the sense of achievement and satisfaction of learning but also improve general skills and better achieve knowledge, ability, and emotional goals. Course content quality has no significant effect on online learning engagement (*β* = 0.124, *P* > 0.005). Through communications and interviews with students, blind course section and the improper course selection phenomenon are existed. As a result, students have less course engagement or even drop the course in the midterm. These are the main reasons for the low completion rate of online general course. Online learning experience has a significant positive impact on both online learning engagement (*β* = 0.493, *P* < 0.001) and online learning performance (*β* = 0.484, *P* < 0.001). This indicates that good online learning experience can help students build a sense of self-worth, belonging, realize high-level cognitive activities, and improve learning performance. Online learning engagement has a significance positive effect on learning performance (*β* = 0.671, *P* < 0.001). This result indicates the positive attitude of learning engagement is an important cornerstone and guarantee for achieving excellent learning performance.

### 4.4. Effect Analysis

This section mainly analyzes the interaction mechanism between course content quality, online learning engagement, online learning experience, and online learning performance by total effect, direct effect, and indirect effect of the variables.

#### 4.4.1. Overall Effect and Direct Effect Analysis

The total effect results between each variable in the modified structural model are shown in Table 7. Online learning engagement only has a direct effect on online learning performance (*β* = 0.311), indicating that the continuous and positive state displayed by students during learning is especially critical to achieve an excellent grade. The degree of total effect of online learning experience on each factor from high to low is online learning performance (*β* = 0.637) and online learning engagement (*β* = 0.493). And, it only has a direct effect on online learning engagement. This indicates that a successful online learning experience, such as learning community, input and output, and learning support and service can help in reinforcing learning interest and motivation and getting a good grade by behavioral externalization. The degree of total effect of course content quality on each factor from high to low is online learning performance (*β* = 0.968), online learning experience (*β* = 0.724), and online learning engagement (*β* = 0.357). And, the total effect on online learning experience only has a direct effect, and the total effect on online learning engagement only has an indirect effect. This indicates that course content's appropriateness, practicality, cutting-edge, thinking, systematic, and fun are important to satisfy a good learning experience. Even if the result of course selection does not meet the expectation, it can also transform experience into self-driving force of learning, stimulate learning motivation, and improve learning achievement.

#### 4.4.2. Medium Variables Effect Analysis

In the intervening effect variable analysis, the most used intervening effect value is the ratio of indirect effect by total effect. In this section, there are two intervening variables: online learning engagement and online learning experience (Table 8). In the intervening variable of online learning engagement, online learning performance changes by 0.637 standard deviations when online learning experience changes one standard deviation. Among these, online learning experience influences online learning performance through the intervening variable online learning engagement when effect value is 0.153. However, when effect value is 0.484, online learning experience has a direct effect on online learning performance. The intervening effect accounted for 24.02%, and this indicates the online learning engagement is a significant factor for the online learning performance. However, it is not the key role. In the intervening variable of online learning experience, online learning performance changes by 0.968 standard deviations when content quality changes one standard deviation. Among them, 0.461 indicates the content quality influences online learning performance through the intervening variable online learning experience. However, the remaining 0.507 indicates the content quality has a direct impact on the online learning performance. The intervening effect accounted for 47.62%, which closes to the standard of important influential intervening variable, and this indicates the need to actively improve learning experience, motivate students to adopt in-depth learning ways, and improve learning performance in the online learning process.

#### 4.4.3. Online Learning Performance Effect Analysis

As shown in Figure 4, from the perspective of total effect, the degree of effect of each factor on online learning performance from high to low is course content quality, online learning experience, and online learning engagement. From the perspective of direct effect, the degree of effect of each factor is consistent with total effect. From the indirect effect, the direct effect of curriculum content quality is higher than the intervention effect of e-learning experience. This result shows the key to the online learning performance of the online general course is course content quality and online learning experience. High-quality, satisfying, and demanding teaching content can enable learners to gain a high-level experience, spend more time and energy, and gain more.

## 5. Suggestions

### 5.1. Value the Effect of Course Content

Course content quality is the embodiment of course value. The result of this study revealed the course content quality plays a decisive role on the online learning performance of online general course. Additionally, the perceptual impact of content appropriateness is the most significant one. In another word, the course content should highly fit the learning goals. Therefore, firstly, set up “general education introduction course” for students to understand school's general education objectives, course system, courses selection strategy, and how to deal with general education, etc. Also, developing general literacy test and evaluation helps the students effectively understand their general literacy's advantage and disadvantage, gain personalized resource that can effectively remedy their shortcomings, and further guide course selection to fit their own learning goals. Secondly, value the thinking and cutting-edge facts in the course content when develops and introduces online general courses. Focusing on learning objectives, this paper discusses the evaluation value of learners' perspective in content perception. Moreover, design and research relevant quality analysis tools in order to improve the quality of curriculum content.

Carrying out a separate, specialized and normalized, precise online general course content quality evaluation comprehensively assesses the fitness and effectiveness of existing course and general literacy training in school. Sort by category on a basis of survival of the fittest, building “high-quality” general courses, establishing, and improving a general education course system that meets the quality requirements of the school's students. Practically improve teaching quality of general courses. For example, starting from the goal of talent training and actual school situation, Tianjin University explored a school-based course operation mode from various aspects such as course selection recommendation, process control, assessment setting, test paper customization, and teaching assistant. Lanzhou University used the general literacy assessment to grade the learning difficulties of the courses, let students “check their seats,” scientifically evaluated the implementation effect of general education and made timely adjustments. Sanjiang College took courses and activities as the starting point and constructed a “closed-cycle” application-oriented general education system in colleges and universities of “general course system + classic reading system + series of activities + cultural infiltration.”

### 5.2. Focus on the Medium Effect of Online Learning Experience and Engagement

Results show that the online learning experience can not only directly affect online learning performance but also indirectly affect online learning performance through content quality as a key intervening variable. The most influencing factors on online learning experience are social interaction and evaluation methods. Therefore, firstly, the teachers should guide the students to participate in group discussion, learning, communication, sharing, strengthening their social connections, building a modular and diversified learning community for collaborative learning, and creating learning atmosphere of mutual assistance, mutual learning, and continuous interaction. The cultivation of a good learning community is of great significance to promote the general education, the students' overall training, and the teachers' growth. Secondly, according to course characteristic, clearly defining evaluation methods, designing a scientific course evaluation scale, adopting a multilevel and multitype dynamic assessment mode to evaluate students' comprehensive qualities comprehensively and objectively such as knowledge, abilities, and personal sentiments. Pay more attention to usual performance rather than test scores so that the students can truly enjoy general education.

The experimental results show that online learning investment not only directly affects online learning performance but also indirectly affects online learning performance through learning experience. The most influencing factors for online learning engagement are emotional engagement and cognitive engagement. Therefore, consideration of emotional elements is required while designing the course. Perform emotional design around sensory interaction, behavioral experience, and inner thinking to realize the intervention of learning, thereby promoting student's in-depth learning. In terms of cognitive engagement, using learning analysis technology to collect the feature vector of learner's personality cognition. Design different learning paths, recommending personalized resources and services. The cognition and attitude of learners towards general education are important factors affecting implementation and quality of general education. Good general education should be established on this foundation and try its best to promote students' understanding and cognition towards general education; let them deeply understand the true value and significance of general education, to actively study and grow.

## 6. Conclusion

This paper takes online learning experience, online learning participation, course content quality, and online learning performance as the input layer of neural network and establishes the learning evaluation system of network general education course based on the BP neural network model. This study was based on the 3P model “Presage-Process-Product,” a structural equation model was applied to analyze the structural and effect relationship among learning experience, learning engagement, and learning performance in the online general course. We found that the course content quality is the key factor on analyzing and predicting the early stage and product of learning, and it has the greatest impact on online learning performance. Appropriateness and thinking of content are the key factors affecting content quality. Online learning experience is the important factor which directly affects the online learning performance. It acts as a key intervening variable indirectly affects online learning performance through content quality. Social interaction and course evaluation methods are key factors which affect the online learning experience. Online learning engagement can have a direct and positive effect on the online learning performance. Emotional engagement and cognition engagement are key factors that affecting the online learning engagement. The above conclusions have a certain reference meaning for further optimization of learning effect of online general course. The experimental results show that the method proposed in this paper can effectively detect and evaluate the concentration of students in online course learning and analyze the relevant data. In future research, we will further enrich the variables of early stage and learning process from the aspects of general literacy, in-depth learning strategies, and knowledge acquisition, in order to make the learning impact relationship model of online general education curriculum more comprehensive [23]. In addition, we will combine simulation to prove the robustness of the method.

## Figures and Tables

**Figure 1:** Online general course learning influential relationship model.

**Figure 2:** Schematic diagram of online learning impact relationship.

**Figure 3:** BP neural network model structure for analyzing the relationship between learners, learning process variables and learning performance.

**Figure 4:** Online learning performance factor's performance.

**Table 1:** Operation data for online general course in Zhejiang Shuren College.

Semester	Course number	Course selection number	Pass rate (%)	Excellent rate (%)

Spring 2021	371	18836	88.67	71.46
Fall 2020	366	18745	89.86	71.38
Spring 2020	369	15184	86.29	68.96
Fall 2019	12	8278	92.81	71.92

**Table 2:** Examples for survey item design and references.

1^st^ dimension	2^nd^ dimension

Online learning experience	Social interaction, support and service, evaluation method, input and output, teaching method [21]
Course content quality	Appropriateness, scientific, thinking, balance, fun, cutting-edge [12, 22]
Online learning engagement	Behavioral, cognitive, and emotional engagement, learning motivation [11]
Online learning performance	Self-efficacy, knowledge goals, ability goals, emotional goals, learning satisfaction [22]

**Table 3:** Measurement model's reliability test results.

Latent variable	Average	Standard deviation	Cronbach's *α* value	Average variance extracted (AVE)	Combination reliability (CR)

Course content quality	3.899	0.674	0.869	0.8419	0.8696
Online learning experience	3.819	0.751	0.913	0.7759	0.8453
Online learning engagement	3.618	0.802	0.840	0.7518	0.9135
Online learning performance	3.900	0.681	0.872	0.8665	0.8701

**Table 4:** Measurement model's validity test results.

Latent variable	Observed variable	Factor load	KMO	Approximate Chi-square and *P*	Eigenvalue	Cumulative variance explained rate (%)

Curriculum content quality	Appropriateness	0.874	0.892	874.048 (*P* < 0.000)	4.329	72.148
	Practicality	0.833				
	Cutting edge	0.840				
	Thinking	0.842				
	Systematicness	0.826				
	Fun	0.819				

Online learning experience	Social interaction	0.838	0.811	617.918 (*P* < 0.000)	3.321	71.424
	Input and output	0.784				
	Learning support and service	0.803				
	Evaluation methods	0.816				
	Teaching methods	0.811				

Online learning investment	Behavioral investment	0.846	0.844	595.826 (*P* < 0.000)	3.471	69.772
	Learning motivation	0.774				
	Cognitive investment	0.848				
	Emotional investment	0.893				

Online learning performance	Learning satisfaction	0.927	0.879	727.379 (*P* < 0.000)	3.707	74.136
	Self-efficacy	0.894				
	Knowledge goals	0.891				
	Ability goals	0.866				
	Emotional goals	0.917				

**Table 5:** Discriminative validity results.

	Course content quality	Online learning experience	Online learning engagement	Online learning performance

Course content quality	0.842			
Online learning experience	0.433	0.776		
Online learning engagement	0.394	0.383	0.752	
Online learning performance	0.429	0.413	0.433	0.867
Square root of AVE	0.918	0.881	0.867	0.931

**Table 6:** Model parameter test values and research hypothesis testing results.

	S.E.	C.R.	*P*	Hypothesis testing

H1 Content quality ➔ learning experience	0.059	11.798	^*∗∗∗*^	Yes
H2 Content quality ➔ learning engagement	0.123	0.203	0.839	No
H3 Content quality ➔ learning performance	0.111	4.267	^*∗∗∗*^	Yes
H4 Learning experience ➔ learning engagement	0.142	3.634	^*∗∗∗*^	Yes
H5 Learning experience ➔ learning performance	0.096	5.217	^*∗∗∗*^	Yes
H6 Learning engagement ➔ learning performance	0.514	3.729	^*∗∗∗*^	Yes

Note:  ^*∗*^ ^*∗*^ ^*∗*^*P* < 0.001;  ^*∗*^ ^*∗*^*P* < 0.01; and ^*∗*^*P* < 0.05.

**Table 7:** Total effect values between variables.

Dependent variable independent variable	Online learning experience	Online learning engagement	Online learning performance

Online learning engagement			0.311
Online learning experience		0.493	0.637
Course content quality	0.724	0.357	0.968

**Table 8:** Intervening effect between online learning engagement and online learning experience.

Intervening variable	Path	Effect value	Percentage (%)

Learning engagement	Learning experience ➔ learning performance	0.484	75.98
	Learning experience ➔ learning engagement ➔ learning performance	0.153	24.02

Learning experience	Content quality ➔ learning performance	0.507	52.38
	Content quality ➔ learning experience ➔ learning performance	0.461	47.62

## Data Availability

The data used to support the findings of this study are available upon request.
